# Analysis of the Efficacy and Safety of Pulpitis Treated with Different Root Canal Flushing Fluids Based on VAS and Temporomandibular Joint Function

**DOI:** 10.1155/2022/1470389

**Published:** 2022-08-26

**Authors:** Jianguo Ke, Qiaoling Cai, Churen Zhang, Ou Du, Feixiang Wang, Yu Luo, Wenjin Li, Dongchen Ou

**Affiliations:** Department of Stomatology, The First Affiliated Hospital of Xiamen University, Xiamen 361003, China

## Abstract

Pulpitis is one of the common diseases indicated by the department of stomatology that is located in the tooth and contains abundant nerve vessels. In order to evaluate the pain degree and functional recovery of patients after treatment by visual analogue pain scale (VAS) and temporomandibular joint function score, a retrospective analysis was performed on 128 patients diagnosed with pulpitis who received root canal treatment in the department of stomatology from January 2020 to March 2021. The results show that 3%NaClO combined with 0.9% sodium chloride injection can effectively relieve the pain degree of patients after treatment, and the antibacterial effect is significantly better than 3%H_2_O_2_ combined with 0.9% normal saline. Meanwhile, it can effectively improve the temporomandibular joint function and reduce the recurrence rate, which has good clinical application value.

## 1. Introduction

Pulpitis is one of the common diseases in stomatology, which is often secondary to hard tissue diseases such as caries and wedge-shaped defects and has not been treated in time [1]. In clinical practice, pulpitis patients usually show sudden pain without external stimulation. In severe cases, severe pain will occur when eating hot food, which can only be relieved by gargle and cold water, causing serious harm to both the body and mind of patients [2]. There is a consensus on the pathogenesis of pulpitis in clinical practice, and research has shown that pulpitis is a series of symptoms that manifest themselves under the action of different pathogenic stimuli while the body's resistance is weak, and the ease of the disease depends mainly on the body's resistance, if the body's resistance is strong, pulpitis develops slowly. In this process, removing pathogenic stimuli in time can restore the pulp to health. However, weak resistance of the body will lead to poor local drainage, and the inflammatory exudate is not easy to drain, leading to increased pressure in the medullary cavity, resulting in severe pain [3, 4]. At this stage, different treatment methods are adopted for different stages of pulpitis. For mild pulpitis, it is only necessary to pay attention to oral hygiene and improve body resistance, while for pulpitis caused by dental caries, the tooth should be preserved after root canal treatment to clean up the bacterial infection in the pulp cavity. In the process of root canal treatment, root canal flushing fluid not only has the function of flushing and lubrication but also has certain sterilization and disinfection effects, which are one of the important steps in the process of root canal preparation [5]. Currently, common root canal flushing solutions in China include normal saline and hydrogen peroxide, and sodium hypochlorite (NaClO) is commonly used in foreign countries. However, there are relatively few studies on the effect of NaClO combined with normal saline on root canal flushing in patients with pulpitis in China. Therefore, the study retrospectively analyzes 128 patients who are diagnosed with pulpitis and received root canal therapy in the department of stomatology in our hospital from January 2020 to March 2021 to explore the pain degree, changes in temporomandibular function, and clinical efficacy of NaClO combined with normal saline in these patients after treatment, in order to provide new ideas and theoretical basis for the treatment of pulpitis. It will be reported as follows [6].

The rest of this paper is organized as follows: Section 2 discusses relevant literature and comparative analysis, followed by the clinical treatment methods and evaluation indicators in Section 3. The comparative analysis and data statistics are described in Section 4.  Section 5 concludes the paper with summary and future research directions.

## 2. Related Work

At present, root canal therapy is the main treatment for pulpitis, and root canal flushing is one of the most important steps in the treatment process, especially in the selection of flushing fluid [7]. Brignardello indicated that root canal flushing solution can not only produce chemical effects on pulp tissue to achieve the antibacterial effect in root canal therapy but also timely discharge the inactive pulp and surrounding tissues and bacteria after root canal preparation, thus further reducing the number of bacterial colonies in dental pulp [8]. According to Chandler and Chellappa, after mechanical preparation of root canals, the necrotic tissues and bacteria adhering to the canal wall are too thick, which can affect the seal between the canal wall and the root canal filling material, so the root canal rinse solution is required to remove the aforementioned substances, but the organic and inorganic dentin components in root canal rinse solutions with different chemical properties must be changed [9]. Currently, the most commonly used root canal rinsing solution in clinical practice is H2O2, which can produce oxygen under the action of blocking dehydrogenase for antibacterial purposes, and the active tissue with foaming effect produced during the oxidation process can also lose its effect on the root canal, but during clinical application, this effect is maintained, it was discovered that its acidic qualities can cause varying degrees of irritation to the patient's periapical tissue, and poor surgery can result in subcutaneous emphysema, which is damaging to the patient's prognosis [10]. Based on this, this study found the therapeutic effect of 3%NaClO combined with 0.9% normal saline in patients with pulp and teeth and compared it with 3%H_2_O_2_ combined with 0.9% normal saline root canal rinsing solution to observe the clinical efficacy of the two root canal rinsing solutions for patients.

The study results show that the two groups after treatment in patients with the degree of pain over time are falling, but in the control group, T1 and T2 time had a significantly higher level of pain group (*P* < 0.05) because inherent H_2_O_2_ acidic nature will, in the process of treatment of patients with dental pulp tissue, produce certain irritation and will cause pain. And, treatment at the end of the two groups of patients with anesthesia fade, the control level of pain is slightly higher than that of group, two groups of patients after treatment 6 h anesthesia has completely faded. However, the pain generated by H2O2 stimulation in the control group must remain; hence, a temporary pain degree increase is adopted by the team. Therefore, pain continues to decline after treatment [11]. The results showed that the number of dental colonies in both groups decreased after treatment, and the number of bacterial colonies in the study group is significantly lower than that in the control group, suggesting that the treatment effect of 3%NaClO combined with 0.9% normal saline as root canal flushing solution for pulpitis patients is better than that of 3%H_2_O_2_ combined with 0.9% normal saline. The author analyzed the reasons for the intake and showed that NaClO, as a root canal rinse with a wide antibacterial spectrum, could react with the fatty acids on the organic tissue membrane in the root canal (saponification) and further dissolve them into fatty acid salts and glycerol to achieve the purpose of dissolving pulp tissues [12]. Other studies have shown that, after NaClO is dissolved in water, it forms HClO and NaOH, in which HClO can combine with amino acids in bacterial proteins to produce chemical reactions in bacteria and induce bacterial death, while NaOH can combine with amino acids in dental pulp tissue cells to produce an integrated reaction, further explaining amino acids. It plays a role in cleaning the infected site of root canal [13]. In addition, from this study on two groups of patients before and after treatment, the CMI after comparison shows that the team after the treatment of temporomandibular joint function is better than the control group. By reducing pain and effectively removing colonies to restore temporomandibular joint function, this method can provide good prognostic results for pulpitis patients.

In addition, from this study on two groups of patients for a 1-year follow-up, the results showed that 1-year team pulpitis in patients with recurrence rate is significantly lower than the control group, but in clinical practice, pulpitis recurrence is influenced by additional factors, such as pulp residue after therapy, poor dietary practices,andimmunity. Therefore, it is impossible to explain the close relationship between recurrence and root canal flushing fluid [14, 15]. In addition, some scholars have pointed out that NaClO has certain toxicity and pungent smell that can stimulate periapical tissues and oral mucosa to a certain extent. If the concentration is not properly controlled, patients will also experience pain and other discomfort [16].

## 3. Clinical Treatment Methods and Evaluation Indicators

### 3.1. Patients and Treatment

A retrospective analysis was performed on 128 patients who were diagnosed with pulpitis in our hospital from January 2020 to September 2021 who received root canal treatment in the department of stomatology. According to their personal wishes, the patients are divided into study group (*n* = 59) and control group (*n* = 69). In the study group, there were 27 female patients and 32 male patients aged 27–41. The average duration is 35.35 ± 7.42 years, and the disease lasted from 1 to 3 years, with an average of 2.18 ± 0.59 years. In the control group, there were 34 female patients and 35 male patients, ranging in age from 25 to 42 years, with an average of 34.98 ± 7.62 years, and the disease course from 1 to 4 years, with an average of 2.29 ± 0.53 years. There is no statistical difference in baseline data between the two groups (*P* > 0.05), indicating comparability.

All the patients enrolled in the research signed informed consent, and the specific content included that the examination method and treatment method adopted in the study are clinically applied safe methods; if you have any discomfort during treatment, please inform your doctor-in-charge on time to decide on the next treatment plan. The whole treatment and observation period is 12 months. Please inform the doctor of your condition change on time. During the treatment, do not use any other drugs or other treatment methods for the disease. If you use them, please inform the doctor. In the process of this study, the original data (including the test sheet) belong to the research group, but we will protect your privacy, no matter when your name will not appear in the public publications, if the relevant departments need, they have the right to use these data; your participation is completely voluntary. You have the right to choose not to participate in this study or to withdraw from it at any time. It does not affect the normal treatment of your disease and your illness, but you hope to complete this study without any special reasons [17, 18].

The inclusion criteria include the following aspects: (1) it meets the clinical diagnostic criteria of pulpitis; (2) complete clinical data and general information; (3) single root canal disease; (4) high treatment compliance. The exclusion criteria include the following aspects: (1) lost visitors; (2) a history of pulp treatment; (3) with congenital or acquired immune system diseases; (4) patients with major organ dysfunction.

#### 3.1.1. Method of Root Canal Therapy

In the control group, 3%H_2_O_2_ combined with 0.9% normal saline is used for root canal flushing solution for root canal treatment. Specific procedures are as follows: before treatment, the lesion site is confirmed according to the results of dental films taken by patients, and appropriate root canal working length is determined [19]. The patients are required to use compound chlorhexidine to gargle 2 times, adopt a semisupine position and use 1% iodophor to disinfect the affected teeth and the surrounding oral mucosa, and use a rubber barrier to separate the affected teeth from other healthy teeth. A high-speed turbine drill is used to remove the decay of the dental teeth, and a tell-split drill is used to open the pulp. After the pulp cavity is exposed, a low-speed ball drill is used to slowly open the pulp top, so that the root canal mouth is fully exposed and a linear path suitable for treatment is formed. Fill the root canal with 0.2 ml 0.9% sodium chloride injection. Insert a sterile paper tip into the root canal until a stop is felt. Take it out for 30s and put sterile paper tip into the centrifugal tube for bacterial culture. The sterile paper tip is inserted into the root canal, and the depth did not exceed the length of the root canal. The root canal is dried and sealed with calcium hydroxide paste. The root canal is filled 7 days later, and the patient is asked to return to the hospital for review 6 months later.

The study group took 3%NaClO combined with 0.9% normal saline as root canal flushing solution for root canal treatment. The specific procedures are the same as the control group. Bacteria are cultured in the same way after rinsing, and patients are asked to return to the hospital for review 6 months later.  Figure 1 is the process of root canal treatment.  Figure 2 is the irrigation procedure.

#### 3.1.2. Colony Culture and Counting

The centrifuge tube with sterile paper tip taken during root canal treatment is shaken for 10s, and the upper suspension is smeared on the Petri dish, which is incubated in an anaerobic blood culture flask at 37 °C for 2 d. After 2 d, 0.5 ml of the culture medium is absorbed with a sampling gun, diluted by 10 times, and inoculated into the Petri dish. The Petri dish is placed in a CO_2_ incubator and incubated at 37°C for 2 days. After 2 days, the number of colonies is calculated.

#### 3.1.3. Visual Analogue Scale (VAS)

This scale is mainly used to evaluate the pain degree of patients. The specific operation is to draw a line with a length of 10 cm on the paper, with one end marked as 0, indicating no pain. The other end is marked with 10, indicating extreme pain, and patients are asked to mark on a straight line according to their own perception of pain. Scores ≤ 3 indicate mild pain and tolerable. A score of 4–6 indicates that the pain has affected sleep but is still tolerable. ≥7 indicates that pain is unbearable and affects daily life.

#### 3.1.4. Frinton's Craniomandibular Index (CMI)

The scale mainly included 4 dimensions, including mandibular movement (MM), joint murmurs (JN), joint pressure examination (JP), and masticatory muscle and related muscle group pressure examination (MP), a total of 41 items. During the examination, each item is scored according to negative and positive points, negative points are 0 and positive points are 1. Temporomandibular joint dysfunction index (DI) = (MN + JN + JP)/26; muscle tenderness index (PI) = MP/28; CMI=(DI + PI)/2; the score ranged from 0 to 1; the lower the score is, the better the temporomandibular joint function is.

### 3.2. Treatment Satisfaction Scale

This scale is prepared by our hospital, and the patients' satisfaction with treatment is investigated by oral inquiry. The satisfaction is divided into very dissatisfied, dissatisfied, general, satisfied, and very satisfied. The treatment satisfaction rate = (satisfied + very satisfied)/number of patients × 100%.

### 3.3. Observation Indicators

VAS score is used to compare the changes of pain in T1, T2, T3, and T4. Temporomandibular dysfunction is compared before and after treatment by friction TMJ function score. The number of dental colonies before treatment and 6 months after treatment is compared. The recurrence of pulpitis is compared during one-year follow-up. The treatment satisfaction rate of the two groups is compared with the satisfaction scale designed by our hospital.

### 3.4. Statistical Processing

SPSS 25.0 statistical software is used for data analysis. Measurement data: normality test is performed on the data first. If the data followed normal distribution and homogeneity of variance, it is represented by mean ± standard deviation. Paired sample *T* is used for testing within the group, and variance comparison is used between groups. *F* test is performed for comparison between multiple groups. Repeated measurement an OVA is used between multiple groups to conduct spherical test. Measurement data are expressed as mean ± standard deviation (*x* ®± *s*). Descriptive statistical analysis is conducted by percentage, and *X*^2^ test is performed. *P* < 0.05 indicates significant difference.

## 4. Comparative Analysis and Data Statistics

### 4.1. VAS Changes of T1, T2, T3, and T4

The pain degree of patients in both groups is alleviated after treatment, and the pain degree of patients in the study group at T2 and T3 stage is significantly lower than that in the control group (*P* < 0.05), and there is no significant difference at other time periods (*P* > 0.05), as shown in Table 1. In Table 1, “*∗*” means that it is compared with T1 (^*∗*^*P* < 0.05), “#” indicates that it is compared with T2 (^#^*P* < 0.05), and “&” means that it is compared with T3 (^&^*P* < 0.05).

In Figure 3, “*a, b, c, and d*” mean that if the same letter is shared between groups, *P* > 0.05 at different time points. “#” indicates that *P* < 0.05 between the two groups compared at the same point.

### 4.2. Changes in Fricton TMJ Function Scores before and after Treatment

After treatment, temporomandibular function improved in both groups, and the improvement of function in the study group is significantly better than the control group (*P* < 0.05), as shown in Table 2.

Figure 4 is the changes in fricton TMJ function scores before and after treatment.

### 4.3. Changes in the Number of Affected Dental Colonies Are Compared before Treatment and 6 Months after Treatment

After treatment, the number of affected dental colonies in both groups are decreased, and the number of affected dental colonies in the study group is significantly lower than the control group (*P* < 0.05), as shown in Table 3.

Figure 5 is the number of affected dental colonies in the research group. In addition, root canal treatment and irrigation are shown in Figure 6.

### 4.4. Comparison of One-Year Follow-Up Recurrence Rates

Follow-up results show that the recurrence rate of pulpitis in the study group is significantly lower than that in the control group (*P* < 0.05), as shown in Table 4.

### 4.5. Comparison of Treatment Satisfaction

The satisfaction survey results show that the treatment satisfaction of the study group is significantly higher than that of the control group (*P* < 0.05), as shown in Table 5.

Figure 7 is the comparison of treatment satisfaction.

## 5. Conclusions

From the paper, we can see that, after treatment, the pain degree in the two groups is reduced, and the pain degree in the study group at T2 and T3 stage is significantly lower than that in the control group (*P* < 0.05). The temporomandibular function is improved in both groups, and the improvement of function in the study group is significantly better than that in the control group (*P* < 0.05). The number of affected dental colonies in the two groups after treatment is lower than that before treatment, and the number of affected dental colonies in the study group was significantly lower than that in the control group (*P* < 0.05). The results show that the recurrence rate of pulpitis in the study group is significantly lower than the control group (*P* < 0.05). The study group (93.22%) is significantly higher than the control group (73.91%) (*P* < 0.05). The above method of using 3% NaClO combined with 0.9% saline as the root canal rinsing solution in endodontic treatment of pulpitis can significantly reduce the pain level of patients after up to 6 hours of treatment and remove dental colonies effectively. It can also have a significant improvement in restoring the function of the temporomandibular joint, which is deserving of clinical application for the above treatment and high patient satisfaction.

## Figures and Tables

**Figure 1:** Root canal treatment.

**Figure 2:** Root canal irrigation.

**Figure 3:** VAS changes of T1, T2, T3, and T4.

**Figure 4:** Changes in friction TMJ function scores.

**Figure 5:** The number of affected dental colonies in the research group.

**Figure 6:** The root canal treatment and irrigation.

**Figure 7:** Comparison of treatment satisfaction.

**Table 1:** Comparison of pain degree.

	Number	T1	T2	T3	T4	*F*	*P*
Control group	69	7.27 ± 1.28	5.21 ± 1.23 ^*∗*^	5.37 ± 1.22 ^*∗*^	2.17 ± 0.41 ^*∗*^^#&^	4.2723	<0.001
Study group	59	7.25 ± 1.26	4.58 ± 1.18 ^*∗*^	3.75 ± 1.04 ^*∗*^^#^	2.18 ± 0.42 ^*∗*^^#&^	4.284	<0.001
*t*		0.089	2.943	8.009	0.136		
*P*		0.929	0.017	<0.001	0.892		

**Table 2:** Comparison of DMI.

	Number	Before treatment	After treatment	*t*	*P*
Control group	69	0.22 ± 0.03	0.15 ± 0.04	11.629	＜0.001
Study group	59	0.21 ± 0.04	0.12 ± 0.03	13.628	＜0.001
*t*		1.613	4.733		
*P*		0.109	＜0.001		

**Table 3:** Comparison of the number of dental colonies.

	Number	Before treatment	After 6 months	*T*	*P*
Control group	69	804.32 ± 72.18	217.43 ± 28.32	62.874	＜0.001
Study group	59	806.23 ± 71.29	103.24 ± 15.23	74.072	＜0.001
*t*		0.150	27.723		
*P*		0.881	＜0.001		

**Table 4:** Comparison of recurrence rates.

	Number	Recurrence	Recurrence rate
Control group	69	10	14.49%
Study group	59	2	3.39%
*t*			4.615
*P*			0.032

**Table 5:** Comparison of treatment satisfaction.

	Number	Very dissatisfied	Dissatisfied	Normal	Satisfied	Very satisfied	Satisfaction rate
Control group	69	0 (0.00%)	8 (11.59%)	10 (14.49%%)	25 (36.23%)	26 (37.68%)	51 (73.91%)
Study group	59	0 (0.00%)	0 (0.00%)	4 (6.78%)	21 (35.59%)	34 (37.63%)	55 (93.22%)
*t*							8.330
*P*							0.004

## Data Availability

The simulation experiment data used to support the findings of this study are available from the corresponding author upon request.

## References

[1] Dou Z., Xu Z., Wang Q. (2022). Mosapride citrate combined with divine qu disinfectant oral liquid for children function dyspepsia and the influence of serum factors. *Journal of Healthcare Engineering*.

[2] Koli B., Chawla A., Logani A., Kumar V., Sharma S. (2021). Combination of nonsurgical endodontic and vital pulp therapy for management of mature permanent mandibular molar teeth with symptomatic irreversible pulpitis and apical periodontitis. *Journal of Endodontics*.

[3] Emanuel R. (2020). Dexamethasone for pulpitis. *British Dental Journal*.

[4] Agnihotry A., Gill K. S., Stevenson III R. G. (2019). Irreversible pulpitis - a source of antibiotic over-prescription. *Brazilian Dental Journal*.

[5] Sadaf D., Ahmad M. Z., Onakpoya I. J. (2020). Effectiveness of intracanal cryotherapy in root canal therapy: a systematic review and meta-analysis of randomized clinical trials. *Journal of Endodontics*.

[6] Leung M. F., Wang J. (2022). Cardinality-constrained portfolio selection based on collaborative neurodynamic optimization. *Neural Networks*.

[7] Fernandes Zancan R., Hadis M., Burgess D. (2021). A matched irrigation and obturation strategy for root canal therapy. *Scientific Reports*.

[8] Brignardello-Petersen R. (2020). Insufficient evidence regarding the effects of ozone when used as a disinfectant in root canal therapy. *Journal of The American Dental Association*.

[9] Chandler N., Chellappa D. (2019). Lubrication during root canal treatment. *Australian Endodontic Journal*.

[10] Mishra L., Khan A. S., Velo M. M. d. A. C. (1967). Effects of surface treatments of glass fiber-reinforced post on bond strength to root dentine: a systematic review. *Materials*.

[11] Ruksakiet K., Hanak L., Farkas N. (2020). Antimicrobial efficacy of chlorhexidine and sodium hypochlorite in root canal disinfection: a systematic review and meta-analysis of randomized controlled trials. *Journal of Endodontics*.

[12] Silva E. J. N. L., Prado M. C., Soares D. N., Hecksher F., Martins J. N. R., Fidalgo T. K. S. (2020). The effect of ozone therapy in root canal disinfection: a systematic review. *International Endodontic Journal*.

[13] Pacheco-Yanes J., Provenzano J. C., Marceliano-Alves M. F. (2020). Distribution of sodium hypochlorite throughout the mesial root canal system of mandibular molars after adjunctive irrigant activation procedures: a micro-computed tomographic study. *Clinical Oral Investigations*.

[14] Gao G., Zhang P., Xu B. (2022). Analysis of bioelectrical impedance spectrum for elbow stiffness based on hilbert–huang transform. *Contrast Media and Molecular Imaging*.

[15] Chaugule V. B., Panse A. M., Gawali P. N. (2015). Adverse reaction of sodium hypochlorite during endodontic treatment of primary teeth. *International journal of clinical pediatric dentistry*.

[16] Verma N., Sangwan P., Tewari S., Duhan J. (2019). Effect of different concentrations of sodium hypochlorite on outcome of primary root canal treatment: a randomized controlled trial. *Journal of Endodontics*.

[17] Gao G., Cao L., Du X. (2022). Comparison of minimally invasive surgery transforaminal lumbar interbody fusion and TLIF for treatment of lumbar spine stenosis. *Journal of Healthcare Engineering*.

[18] Sung Y. T., Wu J. S. (2018). The visual analogue scale for rating, ranking and paired-comparison (VAS-RRP): a new technique for psychological measurement. *Behavior Research Methods*.

[19] Yuen M. C., Ng S. C., Leung M. F. (2021). A competitive mechanism multi-objective particle swarm optimization algorithm and its application to signalized traffic problem. *Cybernetics & Systems*.

